RETRACTED

# Effects of Cardiac Rehabilitation on Cardiac Function and Quality of Life in Patients with Ischemic Nonobstructive Coronary Artery Disease and Diabetes Mellitus

**DOI:** 10.1155/2022/3487107

**Published:** 2022-05-29

**Authors:** Yuan Wen, Xiaoli Zhang, Weiqun Lan, Shimin Zhao, Qiuhuan Qi, Li Yang

**Affiliations:** ^1^Department of Cardiovascular Medicine, Wuhan Hankou Hospital, Wuhan, China 430012; ^2^Department of Nephrology, Wuhan Hankou Hospital, Wuhan, China 430012; ^3^Department of Endocrinology and Hematology, Wuhan Hankou Hospital, Wuhan, China 430012

## Abstract

**Objective:**

To investigate the effect of cardiac rehabilitation on the quality of life in patients with ischemic and nonobstructive coronary artery disease complicated with diabetes mellitus.

**Methods:**

From January 2020 to June 2021, 100 patients with ischemic nonobstructive coronary heart disease complicated with diabetes were randomly divided into the control group (*n* = 50). The routine drug therapy observation group (50 cases) was treated with routine drugs combined with cardiac rehabilitation at 6 months for 1 course. The curative effect, cardiac function, 6 min walking distance (6MWD), cardiopulmonary exercise test (CPFT) index, SF-36 Health Status Survey Scale, and quality of life score were compared between the two groups.

**Results:**

The total effective rate of the observation group was significantly higher than that of the control group (*P* < 0.05). After treatment, there was no significant change in cardiac function and 6MWD in the control group. The left ventricular ejection fraction and 6MWD in the observation group were significantly higher/longer than those before treatment and the control group (all *P* < 0.05). After treatment, the indexes of CPET in the two groups were improved in varying degrees. The forced vital capacity and oxygen uptake of anaerobic valve in the observation group were significantly higher than those in the control group (all *P* < 0.05). After treatment, the scores of the SF-36 in both groups were improved in varying degrees. The physiological function, general health, energy, mental health, and total scores of the observation group were significantly higher than those of the control group (all *P* < 0.05).

**Conclusion:**

Cardiac rehabilitation can significantly improve the cardiorespiratory function, exercise ability, and quality of life in patients with ischemic and nonobstructive coronary artery disease complicated with diabetes mellitus.

## 1. Introduction

American College of Cardiology (ACC)/National Heart, Lung and Blood Institute funded Women's Ischemic Assessment (WISE) study indicated that 60% of patients had evidence of ischemia due to chest pain or noninvasive examination, and coronary angiography showed no obstructive stenosis of the coronary artery. Such diseases with obvious ischemic symptoms without obstructive coronary stenosis are known as ischemia with nonobstructive coronary artery disease (INOCA) [1]. Several studies [2, 3] have found that despite the absence of obstructive coronary stenosis, the incidence of cardiovascular events and all-cause mortality in INOCA patients is significantly higher than in the normal population. Such patients are usually relieved by coronary angiography that there is no coronary artery stenosis, so they do not need specific health management, let alone drug treatment. However, type 2 diabetes is a common chronic metabolic disease that leads to atherosclerosis and subsequent arterial stenosis, which is an independent risk factor for causing or aggravating INOCA. The incidence of INOCA is associated with a decline in quality of life [2, 4]. Patients with these conditions are often repeatedly referred to primary and secondary care, which drives the utilization of health resources and leads to the failure of long-term follow-up for these conditions.

RETRACTED

Cardiac rehabilitation is an indispensable component in the management of cardiovascular diseases. It can fully improve the prognosis of patients with heart disease, effectively improve their quality of life, and reduce the possibility of recurrence, so that patients recover through cardiac rehabilitation after illness [5]. Early intervention of cardiac rehabilitation can improve the prognosis of patients. The contents and forms of cardiac rehabilitation are very extensive, including exercise, health education, nutrition management, blood pressure, blood glucose, blood lipid management, psychological regulation, and lifestyle guidance, but exercise training is the core content in the process of cardiac rehabilitation. The heart recovers. Studies on patients with left main coronary artery stenosis have also confirmed that exercise training has a significant effect on the rehabilitation of patients with left main coronary artery stenosis [6]. As medical concepts change, the idea that bed rest or physical activity restriction is beneficial to heart disease is now gradually recognized and accepted as a safe and effective exercise treatment for heart disease [7]. Therefore, in this study, based on conventional drug therapy combined with cardiac rehabilitation, the effects of cardiac rehabilitation on cardiac function and quality of life of patients with ischemic and nonobstructive coronary artery disease combined with diabetes were studied for 6 months to observe the effect of cardiac rehabilitation on cardiac function and quality of life in patients with ischemic nonobstructive coronary artery disease complicated with diabetes and its effect on quality of life.

RETRACTED

## 2. Methods

### 2.1. Participants

A retrospective analysis was conducted in January 2020 and June 2021 in our hospital for the treatment of ischemic nonobstructive coronary artery disease with diabetes mellitus. The sample size was 100 cases. All patients were confirmed by electrocardiogram, coronary angiography, and glucose tolerance test, which met the clinical diagnostic criteria of ischemic nonobstructive coronary artery disease and diabetes. Patients with infectious diseases such as congenital heart disease, mental disorders, renal failure, ketoacidosis, and hyperosmotic nonketotic coma were excluded. According to different clinical treatment methods, the above two groups were divided into the control group (*n* = 50) and the observation group (*n* = 50). In the control group, there were 25 males and 25 females. The average age was 62.75 ± 7.82 years. The course of diabetes was 1-8 years, with an average course of 5.26 ± 0.57 years. In the observation group, there were 26 males and 24 females. The average age was 63.24 ± 6.12 years. The course of diabetes was 2-9 years, with an average course of 5.08 ± 0.64 years. There was no significant difference in general data between two groups (*P* > 0.05).

### 2.2. Study Protocol

In this study, 50 patients in the control group received routine treatment, namely, smoking cessation and alcohol, low-salt and low-fat diet, self-emotional control, and other health interventions for ischemic nonobstructive coronary artery disease and diabetes, and standardized medication for coronary heart disease and diabetes, so as to help patients strengthen clinical treatment effects. On this basis, the other 50 cases of the observation group of patients with cardiac rehabilitation treatment mode show specific measures as shown as follows: (1) to provide psychological support: during the period of clinical treatment, health care workers need to focus on patients' emotional state changes and timely find the adverse psychological intervention, in order to provide targeted psychological intervention and to help ease the emotional burden. In addition, nursing staff should inform patients of the relevant matters needing attention in cardiac rehabilitation treatment in advance, so that they can make psychological preparations in advance and improve their compliance and cooperation with clinical nursing intervention; (2) cardiac rehabilitation: accompanied by professional cardiac rehabilitation personnel, patients underwent moderate intensity cardiac rehabilitation exercise, including impedance exercise, aerobic exercise, and flexibility training, under the condition of ECG and blood pressure monitoring every week. It is worth noting that patients should be guided to warm up before exercise, and exercise time is appropriate to 30~40 minutes, to avoid excessive exercise and lead to body discomfort; and (3) regular follow-up: after the completion of the corresponding cardiac rehabilitation treatment course, specialized medical staff will carry out regular follow-up to observe the improvement of the patient's disease and prognosis. At the same time, in order to promote the patient's recovery as soon as possible, the treatment plan can be adjusted appropriately to further promote the clinical treatment effect. Aspirin (75-150 mg/d), clopidogrel (75 mg/d) oral dual antiplatelet, atorvastatin calcium (20 mg/d) lipid-lowering, plaque stabilization, angiotensin-converting enzyme inhibitors, angiotensin II receptor antagonists, and other cardiovascular protection.

RETRACTED

### 2.3. Observation Index

(1) Cardiac function index: left ventricular ejection fraction (LVEF), left ventricular end-diastolic diameter (LVEDD), and left ventricular end-systolic diameter (LVESD) were measured by color Doppler ultrasound (Toshiba NemioMX ultrasound instrument). (2) Exercise ability: 6 min walking distance (6MWD) was measured. (3) Cardiopulmonary exercise test (CPET): use the treadmill continuously increasing power scheme (Cardiovit CS-200 Cardiopulmonary function tester of Schiller, Switzerland). The operation procedure is as follows: rest for 3 minutes, empty tread for 3 minutes, and then increase the power by 5-20 W/min according to the patient's age and estimated state to reach the maximum exercise power. The recovery period is 5-10 min. Dynamic monitoring of lung function (including forced vital capacity (FVC), forced expiratory volume in the first second (FEV), maximum air volume (MVV)), respiratory rate, oxygen uptake, and so on. (4) Quality of life: the SF-36 Health Survey was used to evaluate the quality of life. The SF-36 included 36 items in 8 dimensions, including physical function, physical function, physical pain, general health, vitality, social function, emotional function, and mental health. The higher the score, the better the quality of life.

### 2.4. Efficacy Criteria

The obvious effect was that the symptoms disappeared and the heart function improved by grade 2 or above. Effective symptom improvement, heart function improvement grade 1. Ineffectiveness means no significant change, aggravation, or death in cardiac function. Total response rate (%) = (number of effective cases + number of effective cases)/total number of cases × 100%.

RETRACTED

### 2.5. Statistical Analysis

SPSS 20.0 software package was used for data processing. The measurement data were expressed as the *x* ± *s*, and “test” was used for comparison between groups. The *Χ*^2^ test was used for comparison between the counting data groups. *P* < 0.05 was considered statistically significant.

## 3. Results

### 3.1. Comparison of Efficacy between the Two Groups

Both groups completed 6 months of treatment. In the control group, 2 cases were significantly effective, 16 cases were effective, and 32 cases were ineffective; the total effective rate was 36.0% (18/50). In the observation group, 7 cases were significantly effective, 25 cases were effective, and 18 cases were ineffective. The total effective rate in the observation group was 64.0% (32/50). The total effective rate of the observation group was significantly higher than that of the control group, and the difference was statistically significant (*P* < 0.05).

### 3.2. The Cardiac Function Indexes of 2 Groups Were Compared with 6MWD

Before treatment, there was no significant difference in cardiac function indexes and 6MWD between 2 groups (all *P* > 0.05). After treatment, there was no significant improvement in all indexes in the control group, but the LVEF and 6MWD in the observation group were significantly higher than those before treatment and those in the control group (all *P* < 0.05). See Table 1.

### 3.3. Comparison of CPET Results between the Two Groups

Before treatment, there was no significant difference in CPET indexes between 2 groups (all *P* > 0.05). After treatment, CPET indicators in both groups were improved to varying degrees, with statistical significance (all *P* < 0.05). The data are shown in Table 2.

### 3.4. Comparison of Quality of Life between the Two Groups

Before treatment, there was no statistically significant difference in the SF-36 Scale scores between the 2 groups (all *P* > 0.05). After treatment, the SF-36 Scale scores of both groups improved to varying degrees, and the physiological function, general health, energy, mental health, and total score of the observation group were significantly higher than those of the control group, with statistical significance (all *P* < 0.05). See Table 3.

## 4. Discussion

The purpose of cardiac rehabilitation is to relieve clinical symptoms, improve patients' cardiopulmonary function and quality of life, improve prognosis, and reduce mortality and re-hospitalization rate and is an important part of the treatment of cardiovascular diseases, including INOCA [8, 9]. With the development of rehabilitation medicine in China, nosocomial rehabilitation (phase I) and family rehabilitation (phase II) of cardiac rehabilitation have received the attention of medical staff and patients. According to basic diseases, general health status, and physical condition, this study worked out personalized exercise prescription and rehabilitation plan from four aspects: health education, lifestyle guidance, exercise training, and psychological intervention to guide patients to carry out rehabilitation training in stages and observe its curative effect.

RETRACTED

The results of this study showed that the clinical effective rate of patients in the observation group who received cardiac rehabilitation for 6 months was significantly higher than that in the control group, and the cardiac function of patients was significantly improved, which was also consistent with the significant increase of LVEF in patients. The exercise amount of the 6 min walking test was close to l time of daily activity, which was simple and safe, and was also a commonly used evaluation method. In this study, the 6MWD of the observation group was longer than that of the control group after treatment, indicating that the exercise ability of the patients was significantly improved, which was consistent with literature reports [10]. As a noninvasive test method for comprehensive evaluation of cardiopulmonary function and exercise tolerance, CPET is a real-time recording of multisystem functional activities such as respiration, circulation, and metabolism under a certain increased exercise load [11]. In this study, various indexes of the observation group were improved to varying degrees after treatment, and FVC, oxygen uptake threshold, peak power, and peak oxygen pulse were significantly better than those of the control group. FVC is an important index to evaluate lung function. Peak power can reflect athletic ability. Peak oxygen pulse is a widely used analysis index in CPET, and LVEF is often used as a reliable indicator to predict survival rate and evaluate the effect of cardiovascular rehabilitation. The improvement of the above indicators also indicates that the cardiopulmonary function and exercise ability of patients in the observation group have been significantly improved, which is consistent with the observation group's higher clinical efficiency, and 6MWD is more consistent with that of the observation group. In the SF-36 Scale, the physiological function, general health, energy, mental health, and total score of the observation group were significantly higher than those of the control group, suggesting that the quality of life of patients in the observation group was significantly improved. Khalife-Zadeh et al. included 50 ACS patients from 2013 to 2014 and randomly divided them into the control group and the observation group, with 25 patients in each group [12]. The observation group received phase I and 11 cardiac rehabilitation (phase I was completed in hospital, and phase II was completed at home through a telephone follow-up). It was also found that the scores of all dimensions of SF-36 Scale in the observation group were significantly improved compared with before intervention. The control group had no significant change. In addition to general health and social function, the scores of other dimensions in the observation group were higher than those in the control group. Anchah et al. [13] also reported similar results, and cardiac rehabilitation is effective for ACS patients of different ages. A systematic analysis shows that patients with ACS benefit more from long-term (6 months) cardiac rehabilitation and recommends a focus on home-based phase II cardiac rehabilitation [14].

RETRACTED

It should be pointed out that although exercise training is the core link of cardiac rehabilitation, health education and psychological intervention can improve the cognition of disease, relieve patients' fear and tension, help patients cooperate with exercise training, and improve the effect of cardiac rehabilitation [15]. Some studies believe that obesity management is a key point in cardiac rehabilitation, including the control of body mass index and waist circumference, which need to be achieved through lifestyle guidance [16]. Therefore, attention should be paid to all aspects of cardiac rehabilitation.

In conclusion, the addition of cardiac rehabilitation therapy to conventional drug therapy can significantly improve cardiopulmonary function and exercise ability and improve the quality of life of patients with ischemic nonobstructive coronary heart disease complicated with diabetes.

## Figures and Tables

**Table 1:** Comparison of cardiac function indexes and exercise capacity between the two groups before and after treatment.

Groups	*n*	LVEF (%)	LVEDD (mm)	LVESD (mm)	6MWD (m)
Control group	50				
Before the treatment		41.57 ± 5.28	53.28 ± 5.96	51.63 ± 6.28	285.76 ± 26.86
After the treatment		42.69 ± 4.98	52.75 ± 6.06	51.26 ± 5.79	302.96 ± 29.65
Observation group	50				
Before the treatment		41.78 ± 5.11	54.82 ± 5.69	51.44 ± 5.68	284.36 ± 27.65
After the treatment		49.26 ± 4.88	50.99 ± 5.43	49.65 ± 5.06	358.44 ± 30.26

**Table 2:** Comparison of cardiopulmonary exercise test results before and after treatment.

Groups	Control group		Observation group	
	Before the treatment	After the treatment	Before the treatment	After the treatment
FVC (L)	2.09 ± 0.32	2.11 ± 0.35	2.10 ± 0.28	2.45 ± 0.31
LEV (L)	1.95 ± 0.23	1.99 ± 0.29	1.89 ± 0.26	2.06 ± 0.32
MVV (L)	82.95 ± 8.96	80.45 ± 8.27	83.26 ± 8.65	83.02 ± 7.88
Respiration rate (times/min)	26.85 ± 3.16	24.26 ± 2.83	26.96 ± 3.04	26.24 ± 2.75
Anaerobic threshold oxygen uptake (L/min)	0.69 ± 0.09	0.73 ± 0.12	0.71 ± 0.08	0.89 ± 0.10
Anaerobic threshold load (Mets)	3.36 ± 0.41	3.35 ± 0.52	3.47 ± 0.39	3.86 ± 0.42

RETRACTED

**Table 3:** Comparison of the SF-36 Health Status Questionnaire scores before and after treatment.

Groups	Control group		Observation group	
	Before the treatment	After the treatment	Before the treatment	After the treatment
Physiological function	56.82 ± 7.26	63.86 ± 8.41	56.12 ± 6.27	76.58 ± 7.12
Physical pain	40.32 ± 5.29	43.11 ± 5.07	40.67 ± 5.14	45.26 ± 4.62
General health	36.89 ± 4.69	41.88 ± 4.86	37.26 ± 4.16	53.86 ± 4.95
Energy	47.96 ± 5.36	58.12 ± 6.49	48.03 ± 4.99	69.75 ± 7.08
Social function	63.28 ± 8.19	65.84 ± 7.28	63.39 ± 7.48	69.54 ± 7.82
Emotional function	41.36 ± 6.14	43.68 ± 6.72	40.98 ± 5.28	47.96 ± 5.66
Mental health	55.86 ± 7.88	62.72 ± 8.36	56.03 ± 6.24	78.64 ± 7.38
Total score	339.28 ± 44.56	375 ± 42.34	340.65 ± 38.25	438.95 ± 40.13

## Data Availability

The datasets used and analyzed during the current study are available from the corresponding author upon reasonable request.
